# Effects of Vitamin C Combined with Growth Inhibitors on Gastrointestinal Bleeding in Cirrhosis

**DOI:** 10.1155/2022/5319786

**Published:** 2022-07-18

**Authors:** Shimei Wang, Yuanyuan Peng

**Affiliations:** ^1^Department of Gastroenterology, Zhuji People's Hospital of Zhejiang Province, Zhuji, China; ^2^Department of Gastroenterology, Xinchang County People's Hospital Affiliated to Wenzhou Medical University, Shaoxing, China

## Abstract

The purpose of this study was to investigate the effect of vitamin C combined with growth inhibitors on serum miR-130a, nitric oxide (NO), and hemostasis in the treatment of upper gastrointestinal bleeding (UGIB) in cirrhosis. Eighty patients with cirrhosis UGIB treated in our hospital from March 2021 to March 2022 were selected and divided into two groups using the random number table method. The control group received growth inhibitor treatment, while the observation group was given vitamin C combined with growth inhibitor treatment for 3 d. The hemostatic effect, serum laboratory indexes (miR-130a, NO), liver function indexes (aspartate aminotransferase (AST), alanine aminotransferase (ALT)), adverse effects, and 24 h hemostasis rate were compared between the two groups. The hemostasis time in the observation group was shorter than that in the control group, and the blood transfusion volume was lower than that in the control group. There was no statistical difference regarding the portal blood flow, miR-130a, NO, AST, and ALT indexes between the two groups before treatment. After treatment, the portal blood flow, miR-130a, NO, AST, and ALT indexes in both groups were lower than those before treatment, and all of them were lower in the observation group than in the control group. Adverse reactions showed no significant difference between the two groups of patients with cirrhosis UGIB,, while the 24 h hemostasis rate in the observation group (97.50%) was significantly higher than that in the control group (77.50%). Vitamin C combined with growth inhibitor was effective in the treatment of cirrhotic UGIB, which could effectively shorten the hemostasis time, reduce the transfusion volume and portal blood flow, and improve miR-130a, NO, and liver function levels of patients, with higher safety, and is worthy of clinical promotion.

## 1. Introduction

Cirrhosis is diffuse liver fibrosis caused by chronic liver diseases such as alcoholic liver disease, hepatitis B, and hepatitis C, accompanied by regenerative nodules, resulting in distorted and deformed liver lobules and microvascular structures. The disease imposes a heavy global health economic burden. Studies [1] have reported 1.16 million deaths per year from cirrhosis, with age-standardized mortality rates showing an increasing trend each year. Upper gastrointestinal bleeding (UGIB) is a common high-risk complication of cirrhosis, and its etiology can be divided into esophageal varices (OV) and nonvariceal bleeding. Domestic scholars have reported [2] that the incidence of OV in patients with UGIB has increased from 6.4% to 15.1% in recent years.

Relevant foreign studies [3] reported that OV occupied about 90.60% of patients with cirrhotic UGIB. Once cirrhosis and UGIB are comorbid, it indicates a high risk of entering the decompensated phase and adverse prognostic outcomes such as hemorrhagic shock or death [4]. Some studies have reported [5] that there is a close relationship between the severity of symptoms and the degree of liver function impairment in patients with cirrhotic UGIB and their mortality. Therefore, active treatment of patients with cirrhotic UGIB is clinically considered to be beneficial in improving the quality of their prognosis. In recent years, it has been reported [6] that growth inhibitors have been shown to be effective in the treatment of cirrhotic UGIB because of their ability to stop bleeding and reduce portal hypertension.

It has also been reported [7] that vitamin C is effective in improving the function of endothelial cells in the liver sinusoids and can also be used in the treatment of cirrhotic UGIB. Although the therapeutic effect of vitamin C and growth inhibitors has been clinically proven, the effect of the combination of the two drugs has not been reported, and their therapeutic effect still needs to be further demonstrated. Based on this, this study will analyze the effect of vitamin C combined with growth inhibitor in the treatment of patients with cirrhotic UGIB and the pathway of influence, with the aim of clarifying the advantages of vitamin C combined with growth inhibitor treatment and providing a more ideal treatment strategy for patients. This study was approved by the Ethical Committee of Zhuji People's Hospital of Zhejiang Province. All participants signed the relevant consent forms before the study.

## 2. Patients and Methods

### 2.1. Patients

Eighty patients with cirrhotic UGIB attending our hospital from March 2021 to March 2022 were selected, and the sequence generated by the random number table was divided into two groups of 40 cases each. Inclusion criteria were as follows: (1) patients had a clear previous history of cirrhosis (refer to the Guidelines for the Diagnosis and Treatment of Cirrhosis [8]); (2) patients met the diagnostic criteria for cirrhotic UGIB in the Guidelines for the Prevention and Treatment of Esophagogastric Variceal Bleeding in Portal Hypertension in Cirrhosis [9] (signs of active bleeding from varices were confirmed by endoscopy); (3) patients had stable vital signs and signed an informed consent form. Exclusion criteria were as follows: (1) patients with a previous history of bleeding from varices in the esophagus or a history of liver transplantation; (2) patients with cirrhotic UGIB induced by malignant tumors in the lower gastrointestinal system or by peptic ulcers and other etiologies; (3) patients who were unable to cooperate with the treatment or who were allergic to the drugs used in this study.

### 2.2. Method

Both groups were given conventional treatment, including strategies for hemostasis, restoration of blood volume (depending on the patient's bleeding condition with definite volume expansion and blood transfusion), and liver protection. Meanwhile, the control group was given growth inhibitor (manufacturer: Shenzhen Squire Pharmaceutical Co. Ltd. (Shenzhen, China), specification: 2 mg, State Drug Quantifier: H20064372) treatment, configured with 3 mg growth inhibitor 12 h solution (dissolved in saline), followed by a slow intravenous push of 0.25 mg (equipped with 1 ml saline dissolved), followed by a continuous infusion of 0.25 mg/h. When the bleeding has stopped, the dose is continued for 3 d of continuous treatment. In the observation group, vitamin C (manufacturer: Hubei Qianjiang Pharmaceutical Co. Ltd., specification: 2 ml: 0.25 g, State Drug quantification: H42020663) was given in combination with growth inhibitor. The duration of intravenous drip was 3 d in both groups.

### 2.3. Outcome Measures

The hemostatic effect was compared between the two groups: the hemostatic time, blood transfusion volume, and portal vein blood flow were recorded. Portal vein blood flow was measured by Doppler ultrasound (manufacturer: Samsung Madison Co. Ltd. XW80A). Serum laboratory parameters were compared between the two groups: indicators included miR-130a and NO, and NO levels were measured by indirect colorimetry (kit source: Wuhan EliRuide Biotechnology Co. Ltd., Wuhan, China). Quantitative reverse transcription-polymerase chain reaction (qRT-PCR) (RNA extraction kit source: Invitrogen, GrandIsland, NY, USA) was used to test miR-130a expression, which was strictly performed as required by the kit. Liver function indicators were compared between the two groups: aspartate aminotransferase (AST) and alanine aminotransferase (ALT) were measured using a semiautomatic biochemical detector (manufacturer: Mindray BS230). The adverse reactions and 24 h hemostasis rate were compared between the two groups: the total incidence rate of nausea, vomiting, abdominal distension, palpitation, and other adverse reactions was counted, and the 24 h hemostasis rate (24 h hemostasis patients/total sample size) was counted.

### 2.4. Statistical Analysis

Statistical Product and Service Solutions (SPSS) 23.0 (IBM, Armonk, NY, USA) was applied for statistical analysis. An independent sample *t*-test was used for comparison between groups for measurement data obeying normal distribution, and an independent sample *t*-test was used for comparison within groups, all expressed as ($\bar{x}$ ± *s*). The count data were tested by *χ*^2^ and expressed as rate (%), and rank series were tested by rank-sum (*Z*). *P* < 0.05 indicates a statistical difference.

## 3. Results

### 3.1. Comparison of Baseline Data between the Two Groups

There was no statistically significant difference in the baseline data of cirrhotic UGIB patients between the two groups (*P* > 0.05) (Table 1).

### 3.2. Comparison of Hemostatic Effect between the Two Groups

There was no significant difference in portal vein blood flow between the two groups before treatment (*P* > 0.05) (Table 2); the hemostatic time in the observation group was higher than that in the control group, and the blood transfusion volume and portal vein blood flow after treatment were lower than those in the control group (*P* < 0.05) (Figure 1).

### 3.3. Serum Laboratory Parameters and Liver Function Parameters Were Compared between the Two Groups

Before treatment, there was no significant difference in miR-130a, NO, AST, and ALT indicators between the two groups of cirrhotic UGIB patients (*P* > 0.05); after treatment, miR-130a, NO, AST, and ALT indicators in the two groups were lower than those before treatment, and the observation group was significantly lower than the control group (*P* < 0.05) (Table 3 and Figure 2).

### 3.4. Comparison of Adverse Reactions and 24 h Hemostatic Rate between the Two Groups

There was no significant difference in the adverse reaction rate between the two groups (*P* > 0.05), while the 24 h hemostasis rate in the observation group (97.50%) was significantly higher than that in the control group (77.50%) (*P* < 0.05) (Table 4).

## 4. Discussion

The pathogenesis of cirrhosis UGIB is mainly related to cirrhosis portal hypertension, impaired liver function, coagulation-anticoagulation mechanism disorders, and portal vein internal diameter, when cirrhosis continues to progress into the decompensated stage, it will destroy the normal liver blood sinusoidal structure and function, affecting the portal blood return, prompting the tissue pressure to increase, the internal diameter due to blood stasis widening, forming the esophagogastric fundus. The more severe the injury, the more serious the destruction of the normal structure of the blood sinusoids will be, leading to the accumulation of blood in the upper gastric collateral circulation and the formation of esophageal varices and the occurrence of UGIB [10]. For patients with cirrhotic UGIB, clinical treatment principles are based on hemostasis and reduction of portal vein pressure, prevention and control of complications, and prolongation of survival, with pharmacological treatment strategies preferred.

Growth inhibitor belongs to the synthetic hormone class (cyclic peptide substances) and is a commonly used clinical hemostatic drug. Its mechanism of action is to regulate the gastrointestinal internal environment, acting directly on the visceral vascular smooth muscle to induce local arterial contraction and reduce its portal blood flow and pressure; by inhibiting the secretion of vasodilating substances (including vasoactive intestinal peptide and substance *P*), it produces local vasoconstrictive effects, and then plays an effective role by inhibiting the secretion of vasodilating substances (including vasoactive intestinal peptides and substance *P*), it produces a local vasoconstrictive effect, which then effectively reduces intestinal vascular resistance and blood flow; at the same time, it can also inhibit the secretion of gastric acid, gastrin, and other irritating substances, which is conducive to repairing the gastrointestinal mucosa [11–13].

Vitamin C is an effective scavenger of reactive oxygen species and has the effect of promoting the formation of antibodies and collagen in the body. Its mechanism of action is to improve the body's immune resistance by participating in amino acid metabolism, neurotransmitters, protein synthesis, and immune function mechanisms; it helps maintain the integrity of blood vessels while reducing the capillary permeability, accelerates blood coagulation, and strengthens hematopoietic function [14]. The results of this study showed that the hemostasis time in the observation group was shorter than that in the control group, and the blood transfusion volume and portal blood flow after treatment were lower than those in the control group (*P* < 0.05). Vitamin C is an important component in the normal biochemistry of the liver and has a high safety profile. It can accelerate blood coagulation and strengthen hematopoietic function by participating in mechanisms such as sugar metabolism and redox; further improving hemostasis efficiency, shortening hemostasis time, reducing blood loss, and lowering transfusion volume. miR-130a is a key factor that regulates gene expression and is involved in the inflammatory response, liver function, and hematopoietic function. It is involved in mechanisms such as inflammatory response and liver function damage [15]. NO is involved in the formation of portal hypertension and hyperdynamic circulation in cirrhotic UGIB and is also closely associated with blood-brain barrier permeability. The abovementioned pathogenesis of cirrhotic UGIB is closely related to the impairment of liver function, and the structure and function of the hepatic blood sinusoids. When liver function is impaired, this results in vitamins synthesised by other organs not being processed and utilised in the liver. Growth inhibitors can inhibit the progression of the disease by improving portal blood flow and pressure and repairing the gastrointestinal mucosa, while the combination of vitamin C can further improve the efficacy of hepatoprotective therapy by multipath intervention. It also improves the level of NO and miR-130a in the liver. There are still limitations in the present study. This is a single-centre study and the conclusions drawn need to be further confirmed by a multicentre, randomized, double-blind study with a larger sample.

## 5. Conclusions

Vitamin C combined with growth inhibitor is effective in the treatment of cirrhosis UGIB, which can effectively shorten the hemostasis time, reduce the transfusion volume and portal blood flow, improve miR-130a, NO, and liver function level of patients, with high safety, and is worthy of clinical promotion.

## Figures and Tables

**Figure 1:** The hemostatic effect was compared between the two groups.

**Figure 2:** Comparison of serum laboratory parameters and liver function parameters between the two groups.

**Table 1:** Comparison of the baseline data of the two groups (*n*, $\bar{x}$ ± *s*).

Group	Number of subjects	Male/female	Age (years)	Etiology of cirrhosis (hepatitis B/alcoholic cirrhosis/hepatitis C)	Child–Pugh classification (A/B/C)	Duration of cirrhosis (years)
Observation group	40	25/15	51.47 ± 6.82	14/15/11	10/14/16	4.39 ± 0.77
Control group	40	27/13	51.74 ± 6.51	16/15/9	9/13/18	4.57 ± 0.71
Χ^2^/*t*/*Z*	—	0.220	0.181	0.333	0.207	1.087
*P* value	—	0.639	0.857	0.846	0.902	0.280

**Table 2:** Comparison of the hemostatic effect between the two groups ($\bar{x}$ ± *s*).

Group	Number of subjects	Hemostasis time (hr)	Blood transfusion volume (ml)	Portal vein flow (mL/min)	
				Post treatment	Before treatment
Observation group	40	17.35 ± 8.74	1091.27 ± 24.31	814.32 ± 93.49	497.38 ± 65.23^*∗*^
Control group	40	22.69 ± 8.31	173.78 ± 29.85	816.17 ± 92.15	604.37 ± 69.48^*∗*^
*t*	—	2.800	11.913	0.089	7.100
*P* value	—	0.006	0.001	0.929	0.001

*P* indicates comparison with that before treatment, *P* < 0.05.

**Table 3:** Comparison of serum laboratory parameters and liver function parameters between the two groups (*n* = 40, $\bar{x}$ ± *s*).

Group	miR-130a		NO (*μ*mol/L)		AST (U/L)		ALT (U/L)	
	Before treatment	Post treatment	Before treatment	Post treatment	Before treatment	Post treatment	Before treatment	Post treatment
Observation group	8.57 ± 1.44	1.79 ± 0.35^*∗*^	124.37 ± 18.95	91.37 ± 10.29^*∗*^	89.48 ± 15.67	20.35 ± 6.74^*∗*^	90.27 ± 16.34	18.64 ± 6.51^*∗*^
Control group	8.51 ± 1.47	2.81 ± 0.37^*∗*^	125.68 ± 18.11	115.67 ± 10.32^*∗*^	88.39 ± 16.14	33.48 ± 6.95^*∗*^	90.11 ± 16.73	32.74 ± 6.87^*∗*^
*t*	0.184	12.666	0.316	10.546	0.307	8.577	0.043	9.422
*P* value	0.854	0.001	0.753	0.001	0.760	0.001	0.966	0.001

*P* indicates comparison with that before treatment, *P* < 0.05.

**Table 4:** Comparison of adverse reactions and 24 h hemostasis rate between the two groups (*n*, (%)).

Group	Number of subjects	Nausea and vomiting	Abdominal distention	Palpitations	Total occurrence	24 h hemostasis rate
Observation group	40	1 (2.50)	1 (2.50)	1 (2.50)	3 (7.50)	39 (97.50)
Control group	40	1 (2.50)	0 (0.00)	1 (2.50)	2 (5.00)	31 (77.50)
Χ^2^	—	—	—	—	0.213	7.314
*P* value	—	—	—	—	0.644	1.7

## Data Availability

The datasets used and analyzed during the current study are available from the corresponding author on reasonable request.
